The article "DICER-dependent biogenesis of let-7 miRNAs affects human cell response to DNA damage via targeting p21/p27" was retracted in 2022. Reasons: manipulated images; original data or images not available; unreliable results or conclusions; concerns about the images.

# DICER-dependent biogenesis of let-7 miRNAs affects human cell response to DNA damage via targeting p21/p27

**DOI:** 10.1093/nar/gku1368

**Published:** 2015-01-10

**Authors:** Bailong Liu, Min Liu, Jian Wang, Xiangming Zhang, Xiang Wang, Ping Wang, Hongyan Wang, Wei Li, Ya Wang

**Affiliations:** 1 Department of Radiation Oncology, The First Hospital of Jilin University, Changchun 130021, China; 2 Department of Radiation Oncology, Emory University School of Medicine and Winship Cancer Institute, Atlanta, GA 30322, USA; 3 Department of Cancer Center, The First Hospital of Jilin University, Changchun 130021, China

## Abstract

Recently, it was reported that knockdown of DICER reduced the ATM-dependent DNA damage response and homologous recombination repair (HRR) via decreasing DICER-generated small RNAs at the damage sites. However, we found that knockdown of DICER dramatically increased cell resistance to camptothecin that induced damage required ATM to facilitate HRR. This phenotype is due to a prolonged G1/S transition via decreasing DICER-dependent biogenesis of miRNA *let-7*, which increased the p21^Waf1/Cip1^/p27^Kip1^ levels and resulted in decreasing the HRR efficiency. These results uncover a novel function of DICER in regulating the cell cycle through miRNA biogenesis, thus affecting cell response to DNA damage.

## INTRODUCTION

MicroRNAs (miRNAs) are ∼22 nucleotide small RNAs that regulate mRNA expression through binding to the 3′ untranslated region (3′UTR) of their target mRNAs. During the miRNA biogenesis process from generating pre-miRNAs to mature miRNAs via digesting the loop off a pre-miRNA, DICER plays a major role (1,2) and a DICER-independent but AGO2-dependent pathway also contributes to the maturation of a few miRNAs, such as miR-451 (3–5). Most human genes are regulated by at least one miRNA (6). Considering that ∼1% of the human genome is devoted to miRNA genes (7), and each miRNA may have many mRNA targets, the potential impact of altered miRNA levels is conceivably enormous. Therefore, miRNAs affect multiple functions of cells through their mRNA targets, which includes affecting cell-cycle distribution and DNA damage response in p53-dependent pathway (8–12) or p53-independent pathway (13–19). Recently, it was reported that the DICER-generated small RNA products at the DNA double-strand break (DSB) sites (20) were required for the ATM-dependent DNA damage response (21) and efficient homologous recombination repair (HRR) (22,23), which was independent of miRNA biogenesis.

Both HRR and non-homologous end-joining (NHEJ) are the two major pathways in mammalian cells to repair DNA DSBs that generated exogenously or endogenously are a severe threat to cell survival. Deficiency in either one of the DNA DSB repair pathways will result in more killing (24,25). Camptothecin (CPT)-induced DSBs at the DNA replication fork (26) require an ATM signaling response (27) to trigger the HRR pathway (28). The reports that DICER was required for the ATM-dependent DNA damage response (21) and efficient HRR (22,23) suggest that knockdown of DICER should sensitize human cells to DNA DSB inducers, particularly to CPT treatment. However, when we examined the effects of knockdown of DICER on the sensitivities of human cells to CPT, we obtained unexpected results: knockdown of DICER made the human cells more resistant to CPT. Through exploring the underlying mechanism, we discovered that knockdown of DICER affecting cell response to DNA damage is independent of the small RNAs but depends on biogenesis reduction of let-7, which results in overexpression of p21^Waf1/Cip1^/p27^Kip1^ and prolonged G1/S transition. Our results provide a new explanation for the effects of DICER on cell response to DNA damage via affecting biogenesis of let-7 to target p21/p27.

## MATERIALS AND METHODS

### Cell lines, irradiation and CPT treatment

The human cell lines used in this study include immortalized fibroblast cell lines MRC5SV (wild type), 180BRM (Lig4 mutant, NHEJ deficient) and AT5BISV (ATM^−/−^, HRR deficient); tumor cells lines HeLa and M059J (DNA-PKcs^−/−^, NHEJ deficient); HRR reporter cells (obtained from Dr. Jasin's lab (29)) and NHEJ reporter cells (obtained from Dr. Pandita's lab (30)). The mouse cell lines used in this study include mouse embryo fibroblast wild-type and Ku80^−/−^ (NHEJ deficient) cells (verified by western blot). These cell lines were grown in Dulbecco's modified Eagle's medium medium supplemented with 10% Fetal Bovine Serum (FBS). The cell irradiation was performed with an X-ray machine (X-RAD 320, North Brandford, CT, USA) at 320 kV, 10 mA with a 2-mm aluminum filter and the dose rate was 2 Gy/min. The cells were treated with CPT that was obtained from NCI at different times before collecting for further detection.

### Construct of FLAG-DICER resistant to siRNA

The plasmid encoding FLAG-hs-DICER was purchased from Addgene. Three rounds of polymerase chain reaction (PCR)-mediated mutagenesis were done on pCAGGS-Flag-hs-Dicer to generate siRNA resistant Dicer1 expression plasmid (Figure 1B) with the proper primers (Supplementary Table S2), which is completely resistant to siGENOME SMARTpool siRNA to human Dicer1. The FLAG control vector was obtained by deleting the Dicer cDNA sequence pCAGGS-Flag-hs-Dicer.

**Figure 1.** Knockdown of DICER causes human cells to become resistant to CPT, a DNA damage inducer. (**A**) MRC5SV and HeLa cells were collected at 60 h after transfecting with control RNA (CtRNA), siRNA pool against DICER (siDICER), FLAG vector, FLAG-DICER or combining transfection. Whole cell lysates were prepared for immunoblot detection. (**B**) Strategy for generating FLAG-DICER construct that is resistant to the pool of siRNA (containing 4 siRNA sequences) against hsa-DICER. (**C**) The effects of knockdown of DICER on cell sensitivity to CPT. MRC5SV and HeLa cells were treated with different concentrations of CPT for an additional 18 h when DICER was knocked down as described in (**A**). The cells were collected for a clonogenic assay. The data presented are the mean and SD from three independent experiments that the authors carried out, *P < 0.05, **P < 0.01. (**D**) Immunoblot detection was performed of ATM^−/−^, M059J or 180BRM cells treated with siDICER as described in (**A**). (**E**) Clonogenic data were obtained from ATM^−/−^, M059J or 180BRM cells treated with CPT (0.1 μM for ATM^−/−^ cells and 0.25 μM for M059J or 180BRM cells) for 18 h when DICER was knocked down as described in (**C**). The cells were collected for a clonogenic assay. The data presented are the mean and SD from three independent experiments that the authors carried out, *P < 0.05.

### siRNAs and transfection

The control RNA and a pool of siRNA against DICER, p21 or p27 were purchased from Dharmacon Inc. Cells were transfected with the plasmid or siRNA for 48–96 h (mouse cells for 30–36 h) then collected for further experiments.

### Cell survival assay

Cell sensitivity to CPT or radiation was evaluated for loss of colony-forming ability. For radiation sensitivity, the cells were exposed to radiation with different doses, and then the cells were collected and plated for colony genesis. For CPT sensitivity, the cells were collected, plated (based on a colony genesis condition) and then treated with different concentrations of CPT at different times; the cells were changed with fresh medium for colony forming. Duplicate dishes were prepared for each dose of irradiation or CPT treatment. The cells were incubated for 10–14 days and the colonies were stained with crystal violet in 100% methanol solution.

### Immonoblotting and antibodies used in this study

The whole cell lyses were prepared as described previously (31). The antibodies against human DICER, DNA-PKcs, Ku70, Lig4, XRCC4, p27/^Kip1^ (also against mouse p27/^Kip1^), CHK1, CHK2, Rad51, Rad54, Cyclin E, Cyclin A, HA, Actin, the mouse DICER and p21^Waf1/Cip1^ were purchased from Santa Cruz Biotechnology Inc. The antibodies against human ATM, Cyclin D1, phosphorylated CHK2 and phospho-histone H3 were purchased from Cell Signaling Technology Inc. The antibodies against autophosphorylated ATM and DNA-PKcs, XRCC2 and XRCC3 were purchased from Abcam Inc. The antibody against Artemis was purchased from Aviva System Biology Inc. The antibody against human p21^Waf1/Cip1^ was purchased from Thermo Scientific Inc.

### Foci of phosphorylated ATM

HeLa cells plated in dishes containing coverslips were treated with control RNA or siDICER for 48 h. The cells were exposed to 2 Gy. At different times, the cells were fixed in 4% paraformaldehyde for 15 min, permeableized for 5 min on ice in 0.2% Triton X-100 and blocked in 10% normal goat serum. The cells on the coverslips were incubated with an anti-phospho-ATM antibody for 3 h at room temperature, washed with 1% bovine serum albumin (BSA) in phosphate buffered saline (PBS) and incubated with an Alexa Fluor 488 goat anti-rabbit LgG(H+L) (purchased from Invitrogen Inc) for 1 h at room temperature. The cells on the coverslips were washed with PBS and mounted using Vectashield-mounting medium with 4′,6-diamidino-2-phenylindole (purchased from Vector Laboratories). Fluorescent images were captured using CarlZeiss Axio Scope A1 with an Epi-Fluorescence microscope equipped with MRm Cooled Digital Camera and Axiovision software (version 4.8) for image acquisition and a module for multichannel display.

### Cell synchronization

To synchronize cells to G1 phase, HeLa cells were cultured in medium without serum for 30 h. To synchronize cells to S phase, HeLa cells were treated with 2 mM thymidine for 16 h and released in 2 h. The cells were collected and the cell-cycle distribution was measured using flow cytometry.

### Cell-cycle distribution, BrdU incorporation and phosph-histone H3 immunostaining

For cell-cycle distribution, HeLa were trypsinized and fixed in 70% ethanol. Cells were then stained in a solution containing 40 μg/ml RNase A, 40 μg/ml propidium iodiden (PI) and 0.1% Triton X-100 in PBS at room temperature for 1 h. The distribution of cells in the cell cycle was then measured using a flow cytometer (Coulter Epics Elite, Miami, FL, USA). For measuring the transition of cells from G1 to S phase, Hela cells were treated with 10 μM BrdU for 45 min at 37°C and 5% CO_2_. The cells were then trypsinized and quenched with media. The precise procedure was followed using BD PharmingenTM BrdU Flow Kits (BD Biosciences, CA, USA). After fixing and permeabilizing the cells with BD Cytofix/Cytoperm Buffer, the cells were incubated with BD Cytoperm Permeabilization Buffer Plus and re-fixed with BD Cytofix/Cytoperm Buffer. The cells were treated with DNase for exposure of incorporated Brdu. The cells were incubated with fluorescent antibodies, resuspended in 1 ml of staining buffer containing 20 μl of 7-AAD solution and analyzed with a flow cytometer. HeLa cells used for the phosphorylated histone H3 immunostaining were fixed in 70% ethanol at −20°C overnight, then permeabilized with 0.25% Triton X-100 at 4°C for 20 min, blocked with 1% BSA and incubated with anti-p-H3 antibody at 4°C overnight. The cells were washed with PBS, incubated with fluorescein isothiocyanate-conjugated Goat Anti-Mouse IgG(H+L) (purchased from STEMCELL Technologies) on ice for 1 h, washed with PBS and stained with PI before analysis using flow cytometry.

### MicroArray of miRNA

MRC5SV cells were treated with control RNA or siRNA against DICER for 60 h. The cells were collected and the RNA was extracted using the miRNeasy Mini kit purchased from Qiagen Inc. The hsa-miRNA expression profile was performed and analyzed by LC Sciences Inc. The assay used 1 μg total RNA samples. The RNA samples were first subject to dephosphorylation reaction to remove 5′ phosphate groups of miRNA molecules. Then an oligonucleotide adapter was added to 3′ end of sample (3′OH containing) RNA sequences using T4 RNA ligase. The adapter sequence contains a tag segment for capturing fluorescent dye during a later dye staining process. Hybridization was performed on a μParaflo™ microfluidic chip using a micro-circulation pump (32). Inside the microfluidic chip, each detection probe consists of a chemically modified nucleotide coding segment complementary to target 2555 unique mature human miRNAs (from miRBase 20, http://www.miRBase.org/) and other RNA (control sequences). The coding segments of the probe molecules were extended away from corresponding substrate surface by polyethylene glycol spacers, which reduced steric hindrance and surface charge effects during hybridization. The probes were synthesized *in situ* using PGR (photogenerated reagent) chemistry (33). Probe/target pair melting temperatures were balanced by chemical modifications and sequence length adjustment to the coding segments of the probes. Hybridization reaction was carried out in 100 μl 6×SSPE buffer (0.90 M NaCl, 60 mM Na_2_HPO_4_, 6 mM EDTA, 25% formamide, pH 6.8) at 40°C overnight. Then the chip was stained using a tag-specific fluorescence dye (Af3 from Invitrogen). Hybridization images were collected using a laser scanner (GenePix 4000B, Molecular Device) and digitized using Array-Pro image analysis software (Media Cybernetics). Data were analyzed by first subtracting background and then, normalizing signals using a LOWESS filter (Locally-weighted Regression) that was applied to spike-in controls.

### Real-time PCR

To detect the mRNA levels of CDKN1A (the p21 gene) and CDKN1B (the p27 gene), a reverse transcription was performed with the total RNA (1 μg) using a SuperScript III First-Strand Synthesis System kit (purchased from Life Technologies Inc) for reverse transcriptase-PCR. Primer sequences for real-time PCR were purchased from Life Technologies Inc. To detect the let-7 levels in cells, a Taqman miRNA reverse transcription kit was used to prepare the products for the real-time PCR.

### Luciferase reporter assay

The total RNA extracted from MRC5SV cells was used as a template for amplifying wild type or mutated at the potential let-7 binding site of p21 3′-UTR (1-1508) or p27 3′-UTR (44-1263) with proper primers (Supplementary Table S3, the primers for wild type of p27 3′-UTR (44-1263) were purchased from GeneCopoeia Inc) and inserted into the psiCHECK^TM^-2 plasmid that was purchased from Promega Inc. A luciferase assay was performed as described in our previous publication (34). Briefly, 293FT cells were transfected with the plasmid (psiCHECK^TM^-2) containing wild type or mutant 3′-UTRs from different genes (p21 or p27) with 50 nM control RNA or hsa-miR mimics in 12-well plates. The cells were harvested 48 h after transfection, the cells were then lysed with a luciferase assay kit (Promega) according to the manufacturer's protocol and measured on a LUMIstar Galaxy luminescent microplate reader (BMG labtechnologies). β-galactosidase or renilla luciferase was used for normalization.

### HRR or NHEJ reporter assay

Cell HRR reporter assay (29) or NHEJ reporter assay (30) were used as described previously. The U2OS HRR reporter cells or 293 NHEJ reporter cells were treated with control RNA, siDICER, siDICER/sip21/p27 or siDICER/let7b mimics for 48 h and then transfected with I-SceI for an additional 48 h. The cells were collected for detecting fluorescent positive cells using flow cytometry.

### Statistical analysis

The statistical significance of comparisons between two groups was determined with Student's *t*-test. *P*-values of less than 0.05 were considered statistically significant. Pearson's correlation analysis was performed with GraphPad Prism 5.

## RESULTS AND DISCUSSION

### Knockdown of DICER causes human cells to become resistant to CPT, a DNA damage inducer

Since it was reported that knockdown of DICER reduced the HRR efficiency (22,23), knockdown of DICER should sensitize cells to CPT since CPT-induced DNA damage requires HRR (28). To study how knockdown of DICER sensitizes cells to CPT, we examined the effects of the knockdown DICER on the sensitivities of human normal (MRC5SV) and tumor (HeLa) cells to CPT. Unexpectedly, knockdown of DICER made the human cells resistant to CPT (Figure 1A and C). To confirm the results we did a rescue experiment by detecting the effects of expressing the siRNA resistant FLAG-DICER on cell sensitivity to CPT when the endogenous DICER was knocked down. The results showed that expression of the siRNA resistant FLAG-DICER when the endogenous DICER was knocked down (Figure 1A and B), the resistance of the cells to CPT was abolished (Figure 1C). These results strongly support that deficient DICER is the major reason for the cell resistance to CPT treatment. These surprising results also suggest that knockdown of DICER may not directly affect ATM signaling and the HRR pathway since the ATM pathway is required to protect cells from CPT-induced killing (27).

To test this hypothesis, we further examined the effects of knockdown of DICER on sensitivity to CPT in additional human cell lines: ATM^−/−^, M059J (with low ATM expression (35) and deficient in NHEJ due to lack of DNA-PKcs expression (36)) and 180BRM (deficient in NHEJ due to mutation of Lig4 mutant (37)) cells. We also examined the effects of knockdown of DICER on sensitivity to ionizing radiation (IR) in 180BRM and M059J, the NHEJ-deficient cell lines. If knockdown of DICER directly affects ATM signaling and HRR, cells without ATM or with low ATM levels should show less change in sensitivity to CPT, and NHEJ-deficient cells should be more sensitive to IR, because mammalian cells require both NHEJ and HRR to repair IR-induced DNA DSBs (25). Knockdown of DICER made all of these cells significantly resistant to CPT (Figure 1D and E) and did not change the sensitivity of the NHEJ-deficient cells to IR (Supplementary Figure S1A and B). These results strongly support our hypothesis that knockdown of DICER does NOT directly affect ATM signaling and the HRR pathway. Mouse cell lines, Ku80^+/+^ (wild-type) and Ku80^−/−^ (NHEJ-deficient) showed similar results (Supplementary Figure S1C and D). These results provide additional support for our conclusion that knockdown of DICER does not directly affect ATM signaling and the HRR pathway.

To explain the CPT resistance in DICER knockdowns, we examined the levels of the key proteins directly involved in HRR (phosphorylated ATM, Rad51, Rad54, XRCC2 and XRCC3) and NHEJ (phosphorylated DNA-PKcs, Artemis, Ku70, Lig4 and XRCC4) in human cells (MRC5SV and HeLa) by knocking down DICER 1 h after exposure to 5 Gy of IR. Knockdown of DICER did not change the levels of the examined repair proteins (Supplementary Figure S1E), which rules out alterations in expression of DNA DSB repair proteins as a cause of resistance to CPT when DICER is knocked down. To further verify this conclusion, we examined the levels of phosphorylated ATM and the extent of ATM foci formation in MRC5SV and HeLa cells with DICER knocked down, at different times after exposure to IR (2 Gy). Knockdown of DICER did not change the levels of phosphorylated ATM or ATM foci formation in these cells (Supplementary Figure S2A and B), which eliminates the possibility that the CPT-resistant phenotype in DICER knockdowns is because of any change in levels or activities of ATM protein.

### Knockdown of DICER prolongs the G1/S transition through up-regulating p21^Waf1/Cip1^ and p27/^Kip1^

We noted that knockdown of DICER transiently reduced the cell number (Figure 2A), which supports that DICER is required for cell proliferation (38). These results led us to further examine the effects of knockdown of DICER on cell-cycle progress since G1 cells are much more resistant to CPT treatment (Supplementary Figure S3A and B). Knockdown of DICER did induce a G1/S block in CPT-treated cells (Figure 2B, Supplementary Table S1A) and irradiated cells (Supplemental Figure S4A) although IR-induced G2 accumulation and G2/M checkpoint response was not affected (Supplementary Figure S4B and C). We then examined the expression levels of p21^Waf1/Cip1^, p27^Kip1^, Cyclin A, Cycin E and Cyclin D1, the proteins that are involved in the G1/S transition (39–42). Knockdown of DICER changed the levels of p21, p27, Cyclin E and A, but not the level of Cyclin D1 (Figure 2C). Knockdown of p21 and p27 reduced the levels of Cyclin A and E (Figure 2D), the consistency of the Cyclin E and A levels depend on the presence of p21/p27 (13,41). More importantly, knockdown of p21 and p27 reversed the extended G1/S transition induced by knockdown of DICER in CPT-treated cells (Figure 2E, Supplementary Table S1B), indicating that the delay of G1/S transition in CPT-treated cells induced by knockdown of DICER is due to an increase in p21 and p27 expression.

**Figure 2.** Knockdown of DICER prolongs the G1/S transition through up-regulating p21^Waf1/Cip1^ and p27/^Kip1^. (**A**) The number of human cells (MRC5SV, HeLa, ATM^−/−^, M059J and 180BRM) was counted at 72 h after the cells were treated with CtRNA or siDICER. The data were obtained from two independent experiments. (**B**) HeLa cells were collected at 60 h after treatment with CtRNA or siDICER. HeLa cells in the G1 and S phases were detected by combining dye from PI, BrdU labeling and flow cytometry as described in the Supplementary Materials. Similar results were obtained from three independent experiments that the authors carried out. (**C**) Immunoblot detection was performed from MRC5SV and HeLa cells treated with siDICER for 60 h. Similar data were obtained from two independent experiments that the authors carried out. (**D**) HeLa cells were treated with siDICER with or without siRNA against p21 or/and p27 (si-p21, si-p27 or si-p21/si-p27) for 60 h, and the cells were collected for immunoblot detection. Similar data were obtained from two independent experiments. (**E**) The effects of si-p21/si-p27 on the G1-S transition in the DICER knockdowns. HeLa cells were collected for detecting G1 and S phase cell distribution as described in B. Similar results were obtained from three independent experiments that the authors carried out.

### Knockdown of DICER upregulated p21^waf1/Cip1^ and p27/^Kip1^ is due to the reduction of biogenesis of let-7

To investigate how knockdown of DICER increased p21 and p27 expression, we examined the p21 and p27 mRNA levels after knockdown of DICER. Knockdown of DICER did not change the mRNA levels of p21 and p27 (Supplementary Figure S5), indicating that knockdown of DICER up-regulates p21 and p27 (Figure 2C) at a post-transcriptional stage. Since p21 can be expressed in a p53-independent manner (43–45), knockdown of DICER in HeLa and MRC5SV that are deficient in p53 could exclude the possibility that such a change in the p21 level is involved in the p53 pathway. These results also suggest that the changes in the p21/p27 level might be due to miRNA biogenesis. Therefore, we compared the miRNA expression profiles of human fibroblast cells (MRC5SV) with or without knockdown of DICER. Among all 2555 detected miRNAs, there were 89 miRNAs with a real count ≥500, and the effects of knockdown of DICER on these miRNA levels are shown in Supplemental Table S2. Among the 89 miRNAs, only some miRNAs decreased their expression levels, which suggests that this cell line (MRC5SV) is relatively resistant to knockdown of DICER. The remaining DICER, after knocking down DICER in MRC5SV cells, may be enough to process the maturation for the rest of the highly expressed miRNAs.

Notably, the expression-reduced miRNAs in DICER knocked down MRC5SV cells include the *let-7* family. The human *let-7* family has 10 members including miR-98 and miR-202 (46). The expression of most members in the *let-7* family including miR-98 in MRC5SV cells was above 1000 in a real count except miR-202 (Supplementary Table S3). Interestingly, knockdown of DICER reduced the expression of all 10 members of the *let-7* family including miR-98 and miR-202 (46) by >30% (Figure 3A, Supplemental Table S3). Knockdown of AGO2 did not change the let-7 levels (data not shown), suggesting that DICER-dependent miRNA biogenesis and AGO2-dependent miRNA biogenesis have different preferred choices that do not completely overlap. To determine whether *let-7* could target p21 and p27, we measured the levels of p21 and p27 in *let-7* mimic-transfected cells. The p21 and p27 levels were dramatically reduced in the cells treated with *let-7b* mimics (Figure 3B), suggesting that p21 and p27 are targets of *let-7*. We then searched for and found the potential binding sites of *let-7* in the 3′UTR of p21 and p27 (Figure 3C). A luciferase reporter assay showed no change in activity when cells were transfected with a control RNA, but luciferase activity was significantly inhibited when cells were transfected with *let-7b* mimics (Figure 3D). This inhibition of luciferase activity was reversed when the key *let-7b* binding site at the 3′-UTR of p21 or p27 mutated (Figure 3D). These results confirm that human p21 and p27 are the direct targets of *let-7b*. Aside from *let-7b*, other members of the hsa-let-7 family could also target p21, p27 or both (Supplementary Figure S6A), suggesting that the *let-7* family regulates the cell cycle through targeting p21/p27. To test this hypothesis, we examined the G1/S transition in cells treated with *let-7b* mimics while DICER was knocked down. The results showed that overexpression of *let-7b* abolished the extended G1/S transition induced by knockdown of DICER (Figure 3E).

**Figure 3.** Knockdown of DICER-upregulated p21^waf1/Cip1^ and p27/^Kip1^ is due to the reduction of biogenesis of *let-7*. (**A**) Fold reduction of the human *let-7* family members from the microArray of miRNAs from MRC5SV cells treated with siDICER compared with the cells treated with CtRNA. Whole RNA was extracted from the cells and 1 μg of RNA was used for miRNA microarray by LC Sciences Inc. (**B**) The effects of *let-7b* mimics on p21 and p27 expression in the cells with or without DICER knockdown. MRC5SV and HeLa cells were treated with control RNA or siDICER with or without *let-7* mimics for 60 h and then the cells were collected for immunoblot detection. (**C**) Description of potential *let-7b* binding sites at the 3′-UTR of p21 (left) or p27 (right). (**D**) Relative luciferase activities were detected in 293FT cells treated with CtRNA or *let-7* mimics at 48 h after transfection with the luciferase reporter vector containing either the wild type 3′-UTR of p21 or p27 (WT) or the 3′-UTR mutated (MT) at the potential binding site for *let-7* (p21: mutated CTACCT to GATGGA; p27: mutated CTACCT to GATGGA). The data presented are the mean ± SD from three independent experiments that the authors carried out, **P < 0.01. (**E**) The effects of *let-7b* on the G1-S transition in DICER knockdowns. HeLa cells were collected for detecting G1 and S phase cell distribution as described in Figure 2B. Similar results were obtained from three independent experiments that the authors carried out.

Murine p21 and p27 are also efficiently targeted by *let-7d* in embryo fibroblasts cells (Supplementary Figure S6B), suggesting that the regulation of the cell cycle through the *let-7* family to target p21/p27 or their homologues might be conservative among species. *Let-7* was first discovered as a key developmental regulator in nematode (47) and was soon thereafter, found in fruit flies and humans (48). The mature form of *let-7* family members and *let-7* binding sequences at the 3′-UTR of p21/p27 homologues among different species are highly conservative across species (Supplementary Figure S6C and D). Although there is no *let-7* in *Arabidopsis* (49), there is a putative ath-miR-5661 binding site at the 3′-UTR of *ick1* (cyclin-dependent kinase inhibitor 1) in *Arabidopsis* (Supplementary Figure S6C and D). We believe that knockdown of DICER in *Arabidopsis* should have a similar effect on the plant cell transition from G1 to S.

### Prolonged G1/S transition results in decreased HRR and cellular resistance to CPT treatment

Next, we addressed whether the extension of the G1/S transition induced by knockdown of DICER is the major reason for cellular resistance to CPT. For this purpose, we examined the effects of overexpressing *let-7b* mimics or inhibiting p21/p27 on the sensitivity of the DICER knockdowns to CPT. Either overexpressing *let-7b* mimics or inhibiting p21 and p27 in the DICER knockdowns abolished the resistance of the cells to CPT (Figure 4A). It has been reported that knockdown of DICER in human U2OS cells with an integrated I-SceI substrate inhibited the HRR efficiency, which is due to a shortage of DICER-dependent small RNAs at the DSB sites (22,23). However, based on the survival data (Figure 4A), we hypothesized that the reduced HRR efficiency in the DICER knockdowns is due to the extended G1/S transition, since it is known that HRR is much more efficient in the S phase versus the G1 phase. To test this hypothesis, we examined the effects of knockdown of DICER on the levels of *let-7* and p21/p27 in the same reporter cells that were obtained from Dr. Jasin's lab (29). The results confirmed that knockdown of DICER also decreased *let-7* expression (Figure 4B) and increased the levels of p21 and p27 (Figure 4C), which is the same in the HRR reporter cells as shown in other human cell lines tested in this study. More importantly, the inhibition of HRR efficiency caused by knockdown of DICER was completely recovered by transfecting the cells with either siRNA against p21/p27 or with *let-7b* mimics (Figure 4D). These results indicate that the decreased HRR efficiency caused by knockdown of DICER is because of the decreased *let-7* biogenesis, which results in overexpression of p21/p27 and a G1/S transition block. Therefore, even though it has been demonstrated that there are DICER-dependent small RNAs at DNA DSB sites (20–23), our results exclude a functional link between these small RNAs and the ATM activation or HRR efficiency.

**Figure 4.** The prolonged G1/S transition results in decreased HRR and cellular resistance to CPT treatment. (**A**) The effects of *let-7b* mimics, si-p21, si-p27 or si-p21/si-p27 on the sensitivities of cells with DICER knockdown to CPT. MRC5SV and HeLa cells were treated with siDICER and with or without *let-7b* mimics, si-p21, si-p27 or si-p21/si-p27 for 60 h. The cells were collected, plated, treated with CPT for an additional 18 h and then used in the clonogenic assay. The data presented are the mean ± SD from three independent experiments that the authors carried out, *P < 0.05, **P < 0.01 versus bar 2. (**B**) The relative level of *let-7b* was detected in the HRR reporter U2OS cells. The cells were treated with CtRNA or siDICER for 48 h and then transfected with I-SceI for an additional 48 h. The cells were collected for RNA extraction and the *let-7b* levels in siDICER treated cells were calculated as a propotion of the *let-7b* level in the cells treated with CtRNA. The data presented are the mean ± SD from two independent experiments that the authors carried out with triple sets for each experiment: **P < 0.01. (**C**) The U2OS HRR reporter or the 293FT NHEJ reporter cells were treated with siDICER with or without, *let-7b* or si-p21/si-p27 for 48 h, the cells were then transfected with I-SceI for an additional 48 h. The cells were collected for immunoblot detection. Similar data were obtained from two independent experiments that the authors carried out. (**D**) HRR efficiency was detected in the U2OS HRR reporter cells treated with siDICER, plus si-p21/si-p27 or let-7 mimics for 48 h. The cells were then transfected with I-SceI for an additional 48 h. The GFP signals of the cells were detected with flow cytometry. The data presented are the mean ± SD from three independent experiments that the authors carried out, *P < 0.05; **P < 0.01. (**E**) After the 293FT NHEJ reporter cells were treated with siDICER, plus si-p21/si-p27 or let-7b mimics for 48 h, they were transfected with I-SceI for an additional 48 h. The fluorescent signals of the cells were detected with flow cytometry. The cell fluorescent (RFP) only upon repair of I-SceI-induced DSBs by NHEJ. The data were obtained from three independent experiments that the authors carried out, *P < 0.05.

DICER stimulated HRR through promoting cells to enter into S phase support that knockdown of DICER decreased the HRR efficiency and resulted in cells becoming sensitive to ultraviolet (UV) exposure (16) since UV-induced DNA damage requests HRR (50). Why knockdown of DICER decreases the HRR efficiency and not change cell sensitivity to IR (Supplementary Figure S1)? We thought that it might be due to knockdown of DICER increasing G1 phase cells that are more efficient for NHEJ (51), which neutralized the effects of decreased HRR on cell survival following IR. To test this hypothesis, we examined the NHEJ efficiency after knocking down DICER. As we expected, knockdown of DICER in the NHEJ reporter cells (Figure 4E) increased the NHEJ efficiency (Figure 4F), and knockdown of p21 or up-regulation of *let7-b* abolished the increased NHEJ efficiency (Figure 4F), which explains the major reason why knockdown of DICER decreased the HRR efficiency but did not change cell sensitivity to IR. Taken together, our results demonstrate that knockdown of DICER induces cell resistance to CPT, which is mediated by decreasing *let-7* biogenesis, reducing the effects of *let-7* on targeting p21/p27 and resulting in an overexpression of p21/p27 and a prolonged G1/S transition. Our results provide a new explanation for DICER in regulating the G1/S transition (Figure 5), which indirectly affects cell sensitivity and response to DNA damage.

**Figure 5.** A model explaining how DICER modulates the cell's response to DNA damage through biogenesis of the *let-7* family members that target p21/p27 to regulate the G1/S transition.

## SUPPLEMENTARY DATA

Supplementary Data are available at NAR Online.

SUPPLEMENTARY DATA
